This article has been retracted.

# Exosomal microRNA-32-5p induces multidrug resistance in hepatocellular carcinoma via the PI3K/Akt pathway

**DOI:** 10.1186/s13046-018-0677-7

**Published:** 2018-03-12

**Authors:** Xiao Fu, Mengjie Liu, Shengyang Qu, Jiequn Ma, Yamin Zhang, Tingting Shi, Hongqing Wen, Yujuan Yang, Shuhong Wang, Jing Wang, Kejun Nan, Yu Yao, Tao Tian

**Affiliations:** 1 Department of Medical Oncology, The First Affiliated Hospital of Xi’an Jiaotong University, No. 277 Yanta West Road, Xi’an, Shaanxi 710061 People’s Republic of China; 2 Department of Respiratory, Third Hospital of Xi’an, Xi’an, Shaanxi 710018 People’s Republic of China; 3 The Third Department of Cardiology, Shaanxi Provincial People’s Hospital, Xi’an, Shaanxi province 710068 People’s Republic of China

**Keywords:** microRNA-32-5p, PTEN, Exosome, Hepatocellular carcinoma, Multidrug resistance

## Abstract

**Background:**

Multidrug resistance is the main obstacle for hepatocellular carcinoma (HCC) treatment. miR-32-5p is involved in HCC progression but its function in multidrug resistance is still unclear. Here we aim to find out the function of miR-32-5p in inducing multidrug resistance and its underlying mechanisms of transforming sensitive cell to resistant cell.

**Methods:**

We detected the expression of miR-32-5p and PTEN in the multidrug-resistant cell line (Bel/5-FU) and the sensitive cell line (Bel7402), HCC and para-carcinoma liver tissues through real-time PCR. Dual-luciferase reporter assay verified PTEN is the target of miR-32-5p. Exosomes from sensitive and multidrug resistant cell line were obtained and confirmed through ultracentrifuge and Nano Analyzer. Gain- and loss-of-function experiments, rescue experiments, a PI3K/Akt pathway inhibitor, an exosome biogenesis inhibitor, and nude mice xenograft models were used to determine the underlying mechanisms of miR-32-5p and PTEN, as well as exosomal miR-32-5p in inducing multidrug resistance in vitro and in vivo.

**Results:**

miR-32-5p was significantly elevated but PTEN was reduced in Bel/5-FU. An inverse correlation between miR-32-5p and PTEN was confirmed in HCC cell lines and patients; moreover, high expression of miR-32-5p and low expression of PTEN were positively associated with poor prognosis. Over-expression of miR-32-5p activated the PI3K/Akt pathway by suppressing PTEN and induced multidrug resistance via exosomes through promoting angiogenesis and epithelial-mesenchymal transition (EMT).

**Conclusions:**

Our study demonstrated that the multidrug-resistant cell, Bel/5-FU delivers miR-32-5p to sensitive cell, Bel7402 by exosomes and activates the PI3K/Akt pathway to further induce multidrug resistance by modulating angiogenesis and EMT.

**Electronic supplementary material:**

The online version of this article (10.1186/s13046-018-0677-7) contains supplementary material, which is available to authorized users.

## Background

HCC is the sixth most common malignancy and the fourth leading cause of cancer-related death worldwide. Chemotherapeutic drugs, such as 5-fluorouracil (5-FU), oxaliplatin (OXA), and gemcitabine (GEM) are traditional systemic treatments for advanced HCC patients, but the treatment efficacy is disappointing. Recently, in advanced cases of HCC, sorafenib has become the only effective systematic therapy; however, the median life expectancy of patients on sorafenib is only one year [1]. Multidrug resistance has become the predominant obstacle for HCC treatment, thus understanding the mechanisms of multidrug resistance and exploring novel therapeutic targets to overcome multidrug resistance is of great importance.

The PTEN/PI3K/Akt pathway contributes to chemoresistance in different types of cancers by regulating proliferation, apoptosis, angiogenesis, EMT, and autophagy [2, 3]. Moreover, we found that overexpression of PTEN sensitizes HCC cells to sorafenib [4]. Although exon mutation of PTEN is associated with tumorigenesis and chemoresistance [5, 6], down-regulation of PTEN is not always associated with the genetic mutation [7]. Indeed, the subtle decrease in gene dosage or protein activity of PTEN, especially via post-transcriptional regulation, is involved in the progression and treatment resistance of HCC [8, 9]. Recently, a miR-PTEN network has been established in a variety of cancers. Increasing evidence shows that PTEN-regulating miRs, such as miR-141-3p [10], miR-29a [11], miR-21 [12–16], miR-19a [17], miR-92a [18], and miR-486 [19] contribute to anti-tumor treatment resistance. However, how the miR-PTEN network promotes multidrug resistance in HCC remains unknown. Through bioinformatics prediction, literature review, and real-time PCR, we found that elevated miR-32-5p was associated with tumorigenesis in different cancer types, including HCC [20–26]. miR-32-5p also contributes to castration resistance, radioresistance and chemoresistance in prostate cancer [27], but its function in promoting multidrug resistance in HCC remains unclear.

Exosomes are circulating membrane-bound nanovesicles secreted form endosomal pathways. They are the most abundant type of extracellular vehicles (EVs) that range in size from 30 to 150 nm, containing RNAs (especially miRNAs), proteins and other bioactive molecules [28]. Recently, exosomes generated from chemoresistant cells have been proven to deliver miRs and transfer malignant phenotype to sensitive cells [29].

Here, we hypothesize that miR-32-5p induces multidrug resistance in HCC via exosomes through the PTEN/PI3K/Akt pathway. To test our hypothesis, we first examined the expression pattern of miR-32-5p and PTEN in a multidrug-resistant HCC cell line Bel/5-FU and in HCC patients. Then, we analyzed the association between miR-32-5p or PTEN and characteristics of HCC patients and the prognostic value of miR-32-5p and PTEN. Next, we used dual-luciferase reporter assay, real-time PCR, and Western blots to determine PTEN is the direct target of miR-32-5p. Afterwards, we performed gain- and loss-of-function experiments and rescue experiments to confirm that miR-32-5p mediates multidrug resistance by targeting PTEN and hyperactivating the PI3K/Akt pathway in vitro and in vivo. Finally, we extracted the exosomes from both the sensitive cell line and the resistant cell line and estimated the role of exosomal miR-32-5p from resistant cell line in promoting multidrug resistance. In conclusion, we found that exosomal miR-32-5p induces multidrug resistance in HCC through the PTEN/PI3K/Akt pathway by promoting angiogenesis and EMT.

## Methods

### Drugs

5-FU (Sigma-Aldrich, MO, USA) was made into an aqueous solution at a concentration of 25 mg/ml and was administered at doses ranging from 1.6 to 5000 μM. OXA (Sanofi, Paris, France) was dissolved in 5% glucose solution to make a stock concentration of 5 mg/ml and was administered at doses ranging from 0.02 to 100 μM. GEM (Lilly SA, Alcobendas, Spain) was dissolved in 0.9%normal saline (NS) to make a stock concentration of 40 mg/ml and was administered at doses ranging from 0.01 to 31.25 μM. Sorafenib (Bayer AG, Berlin, Germany) was dissolved in DMSO to make a stock solution of 314 μM and was administered at doses ranging from 0.1 to 312.5 μM.

Wortmannin (WM; Sigma, MO, USA) was used to suppress the activity of the PI3K/Akt signaling in Bel/5-FU cells. WM was dissolved in DMSO (Sigma, MO, USA) to make a stock solution of 1 mM and was administered at 100 μM for 24 h.

GW-4869 (Sigma, MO, USA) was dissolved in ethanol (Sigma, MO, USA) with a stock concentration of 0.2 mg/mL and then added to the medium of Bel/5-FU with the concentration of 10 μM to suppress the production of exosomes.

### Cell culture, transfection and treatment

#### Cell lines

The sensitive cell line Bel7402 and the resistant cell line Bel/5-FU were purchased from Key GENE Biotech, Nanjing, Jiangsu, China. Bel7402 and Bel/5-FU cells were cultured in RPMI-1640 medium (Gibco, CA, USA) supplemented with 10%fetal bovine serum (FBS; Biological Industries, CA, USA), 100 IU/ml penicillin and 100 μg/ml streptomycin (HyClone, MA, USA) in humidified atmosphere with 5%CO2 at 37 °C. 5-FU was added at a concentration of 20,000 ng/mL to the medium of Bel/5-FU cells.

HEK-293T, SMCC-7721, HepG2, Hep3B, and MHCC97H cell lines were purchased from the Institute of Biochemistry and Cell Biology, Chinese Academy of Sciences, Shanghai, China, and was cultured in DMEM medium (Gibico, CA, USA), supplemented with 10% fetal bovine serum (FBS; Biological Industries, CA, USA), 100 IU/ml penicillin and 100 μg/ml streptomycin (Hyclone, MA, USA) in humidified 5% CO_2_ at 37 °C.

#### Cell transfection

Cells were plated in 6-well or 24-well plates and transfected with 5 or 10 nM miR-32-5p mimics and inhibitor, 5 nM miR-21-5p mimics and inhibitor, siRNA against PTEN, and respective negative control (NC, GenePharma Co. Ltd., Shanghai, China; the sequences are shown in Additional file 1) or PTEN-expressing vector (Generay Biotech Co., Ltd., Shanghai, China) using Turbo-FectTM (Thermo, MA, USA) according to the manufacturer’s instructions as previously described [8]. RNA was extracted 24 h after transfection, and the transfection efficiency was determined by real-time PCR. Protein was extracted 48 h after transfection for Western blots.

#### Drug resistance assays

Five thousand Bel7402, Bel/5-FU or transfected cells were seeded in 96-well plates (6 replicates per condition). After 12 h, 5-FU, OXA, GEM, and sorafenib were added to the 96-well plates. After 48 h, cell proliferation was measured by 3-(4,5-dimethyl-2-thiazolyl)-2,5-diphenyl-2H-tetrazolium bromide (MTT) assay using FLUOstar OPTIMA (BMG Labtech, Offenburg, Germany). All tests were performed in triplicate.

#### Cell apoptosis detection

Cells were harvested 48 h after transfection. Cell apoptosis was detected by an Annexin-V-7AAD Staining Kit (Key GENE Biotech) as previously [8]. All tests were performed in triplicate.

#### In vitro migration and invasion assays

The migration ability was determined by wound healing assay, and the invasion ability was determined by transwell assay; both were conducted as previously described [8]. All tests were performed in triplicate.

### Patient samples and the cancer genome atlas analysis

All protocols were approved by the Ethics Committee of Xi’an Jiaotong University, and informed consent was obtained from all patients before surgery. 44 formalin-fixed, paraffin-embedded (FFPE) HCC tissues and 28 un-paired para-carcinoma liver tissues from patients who underwent surgery for HCC were obtained from the Department of Hepatobiliary Surgery at The First Affiliated Hospital of Xi’an Jiaotong University from January 2011 to February 2013. Upon enrollment, HCC was confirmed in all patients by biopsy or surgical pathology and graded by the American Joint Committee on Cancer (AJCC) TNM staging system. None of the patients had received chemotherapy or radiotherapy before surgery. The exclusion criteria included the presence of severe concomitant diseases, such as cardiovascular disease, immune depression, kidney disease, etc. The clinical characteristics of the patients included in Tab. 1 were collected from the hospital medical records, and registered patients were prospectively followed up until March 31, 2017.

**Table 1:** Correlation between the clinicopathological characteristics and expression of miR-32-5p and PTEN in HCC patients

Characteristics		Number of patients	miR-32-5p expression (Mean ± SEM)	PTEN expression (Mean ± SEM)
Age	< 50	22	210.20 ± 54.50	6.15 ± 2.59
	> 50	22	269.50 ± 51.36	1.34 ± 0.59
Sex	Male	37	262.59 ± 42.58	4.31 ± 1.60
	Female	7	119.65 ± 47.41	0.73 ± 0.57
TNM Stage	I + II	19	142.32 ± 37.58*	7.20 ± 2.956*
	III + IV	25	314.00 ± 55.21*	1.11 ± 0.47*
Tumor size	< 5 cm	13	252.46 ± 64.51	1.74 ± 0.76
	> 5 cm	24	198.01 ± 44.21	4.68 ± 1.96
Death	Alive	19	5.74 ± 0.63***	8.24 ± 2.88*
	Dead	25	310.04 ± 52.32***	0.32 ± 0.13*
HBV infection	No	3	562.55 ± 124.12	0.07 ± 0.02
	Yes	41	216.24 ± 36.64	4.01 ± 1.46
AFP	< 40	9	200.29 ± 79.81	13.26 ± 5.67
	> 40	35	250.02 ± 42.54	3.74 ± 1.36
Complications	Yes	9	251.26 ± 82.66	2.21 ± 1.13
	No	36	239.31 ± 41.25	11.39 ± 7.44

*p < 0.05, ***p < 0.001 by non-parametric Mann-Whitney-Wilcoxon test

The processed expressional data of miR-32-5p and PTEN and the clinical data in the TCGA were downloaded from FIREHOSE Broad GDAC (http://gdac.broadinstitute.org/). And level 3 Illumina RNA-Seq and miRNA-Seq were used for the analysis of PTEN mRNA and miR-32-5p expression, respectively.

### Luciferase gene reporter assay

The 3’-UTR of PTEN or its mutated versions were cloned into the GP-miRGLO Vector (Promega, WI, USA) and were constructed by GenePharma (Shanghai, China). The relative luciferase activity was measured by a Dual-Luciferase Reporter Assay System (Promega, WI, USA) as previously described [8]. All tests were performed in triplicate.

**Fig. 1:** MiR-32-5p induces multidrug-resistance in HCC. **a** Bel/5-FU is resistant to 5-FU, OXA, GEM and sorafenib, n = three independent experiments, *p < 0.05, **p < 0.01, ***p < 0.001 by Student’s *t*-test. 5-FU, 5-fluorouracil; OXA, oxaliplatin; GEM, gemcitabine. **b** Predicted miRs that have complementary binding sites to the 3’-UTR of PTEN through bioinformatics analysis (DIANA, miRDB, and miR org databases). **c** PTEN mRNA is lower expressed in Bel/5-FU. The PTEN level is normalized to the corresponding inner control GAPDH, and the PTEN/GAPDH in Bel7402 cells is set as 1.0-fold, n = three independent experiments, **p < 0.01 by Student’s *t*-test. **d** The expression of PTEN-related miRs in Bel/5-FU. The miRs levels are normalized to the corresponding inner control U6, and the miRs/U6 in Bel7402 cells is set as 1.0-fold, n = three independent experiments, **p < 0.01 by Student’s *t*-test; miR, microRNA. **e** The reversed expression pattern of miR-32-5p and PTEN in HCC cell lines, n = three independent experiments, *p < 0.05, **p < 0.01, ***p < 0.001 by one-way ANOVA test

### RNA extraction and quantitative real-time PCR

Total RNA was extracted from FFPE HCC tissues from patients by using a miRNeasy FFPE kit (QIAGEN, Hilden, Germany) according to the manufacturer’s protocol. Total RNA was extracted from cultured cells or xenograft tumors using Fast200 (Tiangen, Beijing, China), and the isolated total RNA was reverse transcribed using a Mir-X™ miRNA First-Strand Synthesis Kit (Clontech, CA, USA) for miRs and Prime ScriptTM RT Master Mix (Takara, Shiga, Japan) for mRNAs. The relative expression of miR-32-5p, miR-21-5p, miR-19a-3p, miR-92a-3p, miR-486-5p and U6, PTEN, Twist, Snail, and GAPDH mRNA was measured with SYBR® Premix Ex Taq™ II (Perfect Real Time, Takara, Shiga, Japan) as previously described [8]. The specific primer sequences are shown in Additional file 2. The relative fold-changes were determined by the 2^(-ΔΔCT)^ method, and U6 was used as the internal control for miRs, while GAPDH was used as the internal control for mRNA. All tests were performed in triplicate.

### Protein extraction and western blots

Protein extraction and Western blots were conducted and analyzed as previously described [8] with the antibodies against the following: PTEN, N-Cad, and E-Cad (1:1000; Cell Signaling Technology, MA, USA); Akt and phosphorylated-Akt (phosphorylated on S473), Caspase 3 (1:1000; Abcam, CA, USA); P70S6K and phosphorylated-P70S6K (phosphorylated on S371), mTOR and phosphorylated-mTOR (phosphorylated on S2998; 1:1000; Bioworld, Jiangsu, China); CD63, TSG-101, and Flotillin-1 (1:500; Abcam, CA, USA), and human β-actin (1:5000; Transgene, Beijing, China). The blots were quantified by density relative to β-actin, while the phosphorylation of Akt, mTOR, and P70S6K was determined by density relative to total Akt, mTOR, and P70S6K, respectively. All experiments were performed in triplicate.

### Immunohistochemistry (IHC) and microvascular density (MVD)

IHC and evaluation of PTEN, p-Akt, p-P70S6K, p-mTOR, E-cad, N-cad, Ki67, and CD31 were performed as previously described [8, 30]. The MVD was measured as previously described [30].

### Enzyme-linked immunosorbent assay (ELISA)

Supernatant from transfected cells and tumor tissues from the xenografted nude mice were harvested and preserved in − 80 °C and thawed on ice before use. The concentration of VEGF in the supernatant from the transfected cells and tumor tissues from the xenografted nude mice was quantified using a VEGF ELISA kit (NeoBioscience, Guangdong, China) according to the manufacturer’s instructions as previously described [30]. All experiments were performed in triplicate.

### Isolation and confirmation of exosomes

We used ultracentrifuge to isolate the exosomes from Bel/5-FU and a Delsa Nano Analyzer (DelsaNano, Beckman Coulter, Brea, CA, USA) to measure the size and number of exosomes. For exosome isolation and treatment experiments, exosome-depleted medium (by ultracentrifuged over night at 4 °C) was used. For blocking of exosome release, Bel/5-FU cells were treated with GW-4869 (10 μM) or ethanol (as control) for 48 h. For exosome treatment, 5 × 10^5^cells were seeded into 6-well plate with 10%FBS exosome-depleted medium, and 24 h later, exosomes (50 μg/ml) or PBS were added to each well for 48 h.

**Fig. 2:** miR-32-5p targets PTEN and activates the PI3K/Akt pathway. **a** miR-32-5p and its putative binding sites in the 3’-UTR of PTEN. Mutant miR-32-5p binding sites were generated in the complementary site for the seed region of miR-32-5p. **b** Effects of miR-32-5p on luciferase activity in Bel7402, Bel/5-FU, and HEK293T cells carrying the WT and MuT 3’-UTR of PTEN. n = three independent experiments, *p < 0.05 by Student’s *t*-test. **c** The expression of miR-32-5p and PTEN mRNA according to the increasing dose of miR-32-5p mimics and inhibitor by real-time PCR. The miR-32-5p level is normalized to the corresponding inner control U6, the PTEN level is calculated using the corresponding internal control GAPDH and the miRs/U6 or PTEN/GAPDH in Bel7402 cells is set as 1.0-fold. n = three independent experiments, *p < 0.05, **p < 0.01 by Student’s *t*-test. **d**, **e** The expression of PTEN, phosphorylation of Akt, P70S6K, and mTOR according to the dose of miR-32-5p mimics and inhibitor by Western blots; the up- or down-regulation of PTEN replicates the effects of miR-32-5p inhibitor or mimics, respectively, and PTEN-expressing vector or siPTEN reverses the expression of PTEN and phosphorylation of Akt, P70S6K and mTOR in the cells transfected miR-32-5p mimics or inhibitor, respectively. miR-32-5p mimics and PTEN-targeting siRNA rescue the expression of p-Akt, p-P70S6K and p-mTOR after WM treatment. The relative expression of PTEN is normalized to the level of the corresponding internal control β-actin, and the relative expression of p-Akt, p-P70S6K and p-mTOR is normalized to the levels of Akt, P70S6K, and mTOR, respectively. WT, wild-type; MuT, mutant; p-Akt, phosphorylated Akt; p-P70S6K, phosphorylated P70S6K; p-mTOR, phosphorylated mTOR; siPTEN, PTEN siRNA; WM, Wortmannin

### In vivo experiments

Thirty-two 4-week-old male BALB/c nude mice were purchased from Shanghai Experimental Animal Center. The mice were divided into 2 groups, one group (sixteen mice) was subcutaneously injected with 50 μl of 1.0 × 10^6^ Bel7402 cells combined with 50 μl of Matrigel, and the other (sixteen mice) was subcutaneously injected with 50 μl of 1.0 × 10^6^ Bel/5-FU cells combined with 50 μl of Matrigel. When the tumors reached 4 mm*4 mm (two weeks after implantation), the Bel7402 group was divided into two groups (eight mice per group), one injected with agomiR, and the other injected agomiR negative control (NC), while the Bel/5-FU group was also divided into two subgroups (eight mice per group), one injected with antagomiR, and the other injected with antagomiR NC. Three weeks after implantation, each subgroup was randomly divided into two groups (four mice per group), one to receive 5-FU and the other to receive 0.9%NS intraperitoneal (I.P.) once a week for three weeks (Additional file 3A).

To evaluate the effect of Bel/5-FU derived exosomes in vivo, twelve 4-week-old nude mice were firstly subcutaneously injected with 50 μl of 1.0 × 10^6^ Bel7402 cells. When the tumors reached 4 mm*4 mm (two weeks after implantation), they were divided into two subgroups (six mice per group), one was injected with exosomes from Bel/5-FU (100 μg total protein in 100 μL volume), and the other one injected with 100 μL PBS via intra-tumor injection. Three weeks after implantation, each subgroup was randomly divided into two groups (four mice per group), one to receive 5-FU and the other to receive 0.9%NS I.P. once a week for three weeks. Body weight and general condition of the mice were recorded, and the tumor volumes were measured with a caliper three times per week using the formula: volume = length×width^2^/2.

All in vivo protocols were approved by the Institutional Animal Care and Use Committee of Xi’an Jiaotong University.

### Statistics

The data were presented as the mean ± SD. unless otherwise indicated. To verify whether data followed a normal distribution, the Shapiro-Wilk normality test was performed, then an unpaired *t*-test was applied for data followed normal distribution, and non-parametric Mann-Whitney-Wilcoxon test was applied for data followed non- normal distribution. Multiple variable comparisons were done by one-way ANOVA. The Spearman correlation test was used to determine the correlation coefficient (r) and *p*-value for the correlation between the expression of miR-32-5p and PTEN. The association between miR-32-5p or PTEN and clinical characteristics of HCC patients was performed by Fisher’s exact test. The survival curves were calculated by the Kaplan-Meier method and analyzed by the log-rank test.

All analyses were performed with SPSS 19.0 (SPSS Inc., USA). All tests were two-sided, and *p*-values< 0.05 were considered statistically significant. Statistical significances are presented as * according to the following scheme: *, *p* < 0.05; **, *p* < 0.01; and ***, *p* < 0.001.

## Results

### miR-32-5p was elevated but PTEN was reduced in the multidrug-resistant HCC cell line

We used a drug-resistant subtype Bel/5-FU to determine the role of PTEN and PTEN-related miRs in drug resistance. We confirmed that Bel/5-FU cells were resistant not only to 5-FU but also to OXA, GEM, and sorafenib (Fig. 1a). Through bioinformatics analysis (DIANA, miRDB, and miR. org databases) and literature review, we found that miR-32-5p, miR-19a-3p, miR-92a-3p, and miR-486-5p have complementary binding sites to the 3’-UTR of PTEN (Fig. 1b and Additional file 3). We evaluated the expression of PTEN and these miRs by real-time PCR, and we noticed that PTEN was lower-expressed (Fig. 1c), while miR-32-5p, miR-21-5p, miR-19a-3p, miR-92a-3p, and miR-486-5p were all highly-expressed in Bel/5-FU cells (Fig. 1d). Among these miRs, miR-32-5p was of highest expression, and it is conserved among species (*p* < 0.01, Fig. 1d, Additional file 4). In addition, an inverse expression pattern of miR-32-5p and PTEN was observed among HCC cell lines (Fig. 1e).

**Fig. 3:** Reversed correlations of miR-32-5p and PTEN. **a**, **b** miR-32-5p is up-regulated but PTEN is down-regulated in 44 HCC specimens, compared with 28 unpaired para-carcinoma liver tissues. P Ca, paracarcinoma liver tissues. The miR-32-5p and PTEN levels were calculated using the corresponding inner control U6 and GAPDH respectively, **p < 0.01 by non-parametric Mann-Whitney-Wilcoxon test. **c** Reversed correlations of miR-32-5p and PTEN in HCC patients’ tissues, by Pearson’s correlation test. **d-g** High miR-32-5p or low PTEN in 44 HCC patients predicts shorter OS and PFS, by Kaplan**-**Meier analysis. OS, overall survival, PFS, progression-free survival. **h-k** miR-32-5p is up-regulated but PTEN is down-regulated in both paired and un**-**paired HCC and paracarcinoma liver specimens in TCGA dataset. *p < 0.05, **p < 0.01, ***p < 0.001 by non-parametric Mann-Whitney-Wilcoxon test

### Inverse correlation between miR-32-5p and PTEN in clinical HCC samples

To investigate the relevance of miR-32-5p and PTEN in human HCC samples, we used real-time PCR to determine the expression of miR-32-5p and PTEN in 44 HCC samples and unpaired 28 para-carcinoma liver tissues. We found that miR-32-5p was significantly over-expressed (239.85 ± 37.28-fold and 95.64 ± 31.92-fold in HCC and para-carcinoma tissues, respectively, *p* < 0.01, Fig. 2a), but PTEN was significantly lower-expressed (3.74 ± 1.36-fold and 74.29 ± 25.00-fold in HCC and para-carcinoma tissues, respectively, *p* < 0.01, Fig. 2b) in the 44 HCC specimens compared with the 28 para-carcinoma liver tissues. Additionally, a negative correlation between miR-32-5p and PTEN was observed in the 44 HCC tissues (*r* = − 0.306, *p* = 0.044, Fig. 2c).

**Fig. 4:** miR-32-5p promotes multidrug resistance. **a**-**d** Elevated or reduced expression of miR-32-5p induces or inhibits resistance to 5-FU, OXA, GEM, and sorafenib in vitro. siPTEN enhances, whereas PTEN-expressing vector reverses the resistance to 5-FU, OXA, GEM, and sorafenib. Ectopic expression of PTEN in Bel7402 cells transfected with miR-32-5p mimics rescues the resistance to 5-FU, OXA, GEM, and sorafenib, while inhibition of PTEN in Bel/5-FU cells transduced with miR-32-5p inhibitor reverses the inhibition of 5-FU, OXA, GEM, and sorafenib. WM sensitizes Bel/5-FU cells to 5-FU, OXA, GEM, and sorafenib, but miR-32-5p mimics or siPTEN increases multidrug resistance. n = three independent experiments, *p < 0.05, **p < 0.01, ***p < 0.001 by Student’s *t*-test or one-way ANOVA test. **e** Growth curves of xenograft tumors derived from Bel7402 cells injected with agomiR and Bel/5-FU cells injected with antagomiR in response to 0.9%NS or 5-FU. *p < 0.05, by one-way ANOVA test. 0.9%NS, 0.9% normal saline. **f**, **h** IHC staining for Ki67, PTEN, p-Akt, p-mTOR, and p-P70S6K in xenograft tumors; original magnification, 400×; scale bar, 25 μm. p-Akt, phosphorylated Akt; p-P70S6K, phosphorylated P70S6K; p-mTOR, phosphorylated mTOR. **g** The expression of miR-32-5p in xenograft tumors by real-time PCR. The expression of miR-32-5p is normalized to the level of the corresponding internal control U6. *p < 0.05, **p < 0.01 by Student’s *t*-test

Moreover, we used the average fold change of miR-32-5p (239.00-fold) and PTEN (3.74-fold) as thresholds. The Kaplan–Meier survival curve showed that an increased miR-32-5p expression predicted poor survival with shorter overall survival (OS, 28.74 ± 4.51 and 42.84 ± 4.33 months in miR-32-5p high and low groups, respectively, *p* < 0.05) and progression-free survival (PFS, 24.95 ± 3.57 and 42.84 ± 4.33 months in miR-32-5p high and low groups, respectively, *p* < 0.01). These results confirmed the oncogenic role of miR-32-5p in HCC. Additionally, there was a significant correlation of miR-32-5p level with TNM stage and death but not with other clinical features including age, gender, tumor size, HBV infection, complication, and AFP level. In contrast, a decreased PTEN expression indicated poor prognosis with shorter OS (30.85 ± 3.55 months in PTEN low group and un-reached in PTEN high group, respectively, *p* < 0.01) and shorter PFS (28.47 ± 3.19 months in PTEN low group and un-reached in PTEN high group, respectively, *p* < 0.001). In addition, PTEN level was also correlated with TNM stage and death but not with other clinical features (Fig. 2d-g, Table 1).

To better confirm our results, we obtained analyzed data from the Cancer Genome Analysis (TCGA) through FIREHOSE browser and noticed that miR-32-5p(72.48 ± 7.34-fold and 55.31 ± 2.29-fold in HCC and paired para-carcinoma tissues, respectively, *p* < 0.01, Fig. 2h; 71.30 ± 2.64-fold and 55.30 ± 2.29-fold in HCC and un-paired para-carcinoma tissues, respectively, *p* < 0.001, Fig. 2j)is significantly over-expressed but PTEN (10.67 ± 0.14-fold and in HCC and 11.18 ± 0.04-fold paired para-carcinoma tissues, respectively, *p* < 0.01, Fig. 2i, 10.67 ± 0.03-fold and 11.18 ± 0.04-fold in HCC and unpaired para-carcinoma tissues, respectively, *p* < 0.01, Fig. 2k) is lower-expressed in both paired and unpaired HCC and paracarcinoma liver tissues.

The results suggest that the level of miR-32-5p is negatively correlated with PTEN in human HCC samples and that increased miR-32-5p and decreased PTEN are indicative of malignancy in HCC.

### miR-32-5p targets PTEN and activates the PI3K/Akt pathway

Given the inverse expression pattern of miR-32-5p and PTEN, we generated miR luciferase constructs containing the wild-type (WT) or mutant (MuT) 3’-UTR of PTEN (Fig. 3a) and co-transfected HEK293T, Bel7402 and Bel/5-FU cells with miR-32-5p mimics or inhibitor and WT or MuT PTEN 3’-UTR to validate that PTEN is the direct target of miR-32-5p. The relative luciferase activity was markedly reduced in the three cell lines (70.67%, 69.67% and 71.33% in HEK293T, Bel7402 and Bel/5-FU cells respectively) when they were co-transfected with miR-32-5p mimics and miR reporter pMIR-luc-PTEN 3’-UTR-WT. After the binding sites were mutated, the relative luciferase activity was significantly rescued in the three cell lines (101%, 102% and 113.3% in HEK293T, Bel7402 and Bel/5-FU cells respectively) when they were co-transfected with miR-32-5p mimics with miR reporter pMIR-luc-PTEN 3’-UTR-MuT. Moreover, the relative luciferase activity was significantly increased (123.00%, 120.67% and 117.00% in HEK293T, Bel7402 and Bel/5-FU cells respectively) after the cells were co-transfected with miR-32-5p inhibitor and miR reporter pMIR-luc-PTEN 3’-UTR-WT. We also transfected miR-32-5p mimics or inhibitor together with miR reporter pMIR-luc-PTEN 3’UTR-MuT, and the relative luciferase activity remained unaltered compared to that with the co-transfection of mimics or inhibitor NC and reporter pMIR-luc-vector control. These results indicate that miR-32-5p directly targets the 3’-UTR of PTEN (Fig. 3b).

The inhibitory function of miR-32-5p on PTEN was next determined by real-time PCR, and the expression of PTEN attenuated or enhanced with increasing doses of miR-32-5p mimics or inhibitor, respectively (Fig. 3c). Western blots also showed that miR-32-5p mimics could activate the PI3K/Akt pathway similar to the effects of siPTEN and that miR-32-5p inhibitor suppressed the pathway as does the PTEN-expressing vector. Moreover, co-transfection of miR-32-5p mimics with PTEN-expressing vector rescued the PTEN expression and inhibited the activation of the PI3K/Akt pathway caused by the miR-32-5p mimics, but co-transfection of miR-32-5p inhibitor and siPTEN reverses the effects caused by the inhibitor (Fig. 3d).

To further confirm the functional significance of miR-32-5p on the PI3K/Akt pathway, we used wortmannin (WM), a PI3K/Akt pathway inhibitor, to block the PI3K/Akt pathway in Bel/5-FU cells in which the pathway is hyperactivated. Compared with the Bel/5-FU cells treated with DMSO and miR-32-5p mimics NC, the activation of mTOR, P70S6K, and Akt in the Bel/5-FU cells treated with WM and mimics NC was significantly reduced, indicating that WM inhibits the PI3K/Akt pathway. Based on these results, we transfected miR-32-5p mimics or siPTEN to WM-treated Bel/5-FU cells and found that the expressions of phosphorylated-mTOR (p-mTOR), p-P70S6K and p-Akt significantly increased (Fig. 3e). Since both up-regulation of miR-32-5p and down-regulation of PTEN abolished the inhibitory effects of WM on the PI3K/Akt pathway, we concluded that miR-32-5p activates the PI3K/Akt pathway by suppressing PTEN.

### miR-32-5p/PTEN/PI3K/Akt induces multidrug resistance in vitro as well as in vivo

Gain- and loss-of-function experiments were used to assess the miR-32-5p/PTEN/PI3K/Akt pathway in multidrug resistance both in vitro and in vivo.

We transfected Bel7402 and Bel/5-FU cells with miR-32-5p mimics and inhibitor respectively and investigated the role of miR-32-5p in multidrug resistance. As expected, the IC50 values at 48 h after 5-FU, OXA, GEM and sorafenib treatment significantly increased when the cells were transfected with miR-32-5p mimics but significantly decreased when the cells were transfected with miR-32-5p inhibitor (Fig. 4a).

**Fig. 5:** miR-32-5p promotes multidrug resistance through EMT and angiogenesis in vivo. **a** IHC staining for N-Cad, E-Cad, and CD31 in xenograft tumors. Original magnification, 400×; scale bar, 25 μm. *p < 0.05, **p < 0.01, ***p < 0.001 by Student’s *t*-test. N-Cad, N-Cadherin; E-Cad, E-Cadherin; MVD, microvascular density. **b** The expression of VEGF in xenograft tumors. *p < 0.05, **p < 0.01, ***p < 0.001 by Student’s *t*-test. **c** IHC staining for N-Cad and E-Cad in HCC patients’ tissues. Original magnification, 400×; scale bar, 25 μm. *p < 0.05, **p < 0.01, ***p < 0.001 by non-parametric Mann-Whitney-Wilcoxon test

To further confirm that miR-32-5p induces multidrug resistance by targeting PTEN in HCC, we transfected siPTEN and PTEN-expressing vector into Bel7402 and Bel/5-FU cells, MTT results showed that the reduction of PTEN led to multidrug resistance compared with siRNA NC; however, ectopic expression of PTEN reduced multidrug resistance compared with vector control (Fig. 4b).

Moreover, rescue experiments showed that the PTEN-expressing vector rescued the sensitivity of the cells to 5-FU, OXA, GEM, and sorafenib when co-transfected with miR-32-5p mimics, whereas siPTEN enhanced multidrug resistance when co-transfected with miR-32-5p inhibitor (Fig. 4c).

WM was used to verify the function of miR-32-5p in inducing multidrug resistance. WM alone decreased multidrug resistance, compared with DMSO. However, over-expression of miR-32-5p or reduction of PTEN reversed multidrug resistance (Fig. 4d). Thus, we demonstrated that miR-32-5p/PTEN/PI3K/Akt promotes multidrug resistance in HCC in vitro.

Next, we evaluated the effect of miR-32-5p in 5-FU resistance in vivo. In accordance with the in vitro study, the xenograft tumor growth curve and Ki67 (proliferation marker) staining indicated that agomiR promoted 5-FU resistance in the Bel7402 cells injected into nude mice, but antagomiR reversed these effects (Fig. 4e, f, and Additional file 5). After confirming the expression of miR-32-5p in xenograft tumors by real-time PCR (Fig. 4g), IHC staining for PTEN, p-Akt, p-mTOR, and p-P70S6K showed that agomiR activated the PI3K/Akt pathway by suppressing PTEN, while antagomiR inactivated the pathway in vivo (Fig. 4h).

### miR-32-5p/PTEN/PI3K/Akt induces multidrug resistance via angiogenesis and EMT

Since the inhibition of apoptosis is a common cause of resistance to chemotherapy [31] or sorafenib [32], we assessed the apoptosis rate in miR-32-5p mimics- or inhibitor-transfected Bel7402 and Bel/5-FU cells by flow cytometry. Surprisingly, no significant changes in the apoptosis rate or the expression of Caspase 3 were observed among the transfected cells (Additional file 6). An increasing amount of evidence supports that the tumor microenvironment, especially processes such as angiogenesis, plays a crucial role in treatment resistance [33]. Because we observed that the C2 domain of PTEN inhibits xenograft tumor growth in vivo through angiogenesis but not through apoptosis [30], we hypothesized that miR-32-5p modulated multidrug resistance by promoting angiogenesis. Thus, we estimated microvascular density (MVD) in xenograft tumors by using an antibody against CD31, a marker for endothelial cells and evaluated VEGF expression in xenograft tumors. As expected, agomiR elevated MVD, whereas antagomiR reduced MVD (Fig. 5a). In accordance with the MVD, VEGF expression increased in the agomiR-injected tumors (*p* < 0.01) but decreased in the antagomiR-injected tumors (*p* < 0.001, Fig. 5b).

**Fig. 6:** miR-32-5p promotes multidrug resistance through angiogenesis and EMT in vitro. (**a**-**b**) Western blots for the expression of N-Cad and E-Cad in Bel7402 and Bel/5-FU cell lines transfected with miR-32-5p mimics, inhibitor, siPTEN, or PTEN-expressing vector; co-transfected with miR-32-5p mimics and PTEN-expressing vector or miR-32-5p inhibitor and siPTEN; WM-treated Bel/5-FU cell lines transfected with miR-32-5p mimics, siPTEN, or respective NC. The expression of N-Cad and E-Cad are normalized to the level of the corresponding internal control β-actin. **c** Real-time PCR to analyze the expression of Twist and Snail mRNA in Bel7402 and Bel/5-FU cell lines transfected with miR-32-5p mimics, inhibitor, siPTEN or PTEN-expressing vector; co-transfected with miR-32-5p mimics and PTEN-expressing vector or miR-32-5p inhibitor and siPTEN; and WM-treated Bel/5-FU cell lines transfected miR-32-5p mimics or siPTEN. The levels of Twist and Snail mRNA are normalized to the level of the corresponding internal control GAPDH. n = three independent experiments, *p < 0.05, **p < 0.01, ***p < 0.001 by one-way ANOVA test. **d** ELISA for VEGF in the supernatant of Bel7402 and Bel/5-FU cell lines transfected with miR-32-5p mimics, inhibitor, siPTEN or PTEN-expressing vector, co-transfected with miR-32-5p mimics and PTEN-expressing vctor or miR-32-5p inhibitor and siPTEN, and WM-treated Bel/5-FU cell lines transfected with miR-32-5p mimics or siPTEN. n = three independent experiments, *p < 0.05, **p < 0.01, ***p < 0.001 by Student’s *t*-test. **e**-**g** Transwell and wound healing assays in Bel7402 and Bel/5-FU cell lines transfected with miR-32-5p mimics, inhibitor, siPTEN or PTEN-expressing vector, co-transfected with miR-32-5p mimics and PTEN-expressing vector or miR-32-5p inhibitor and siPTEN, and WM-treated Bel/5-FU cell lines transfected with miR-32-5p mimics or siPTEN. n = three independent experiments, *p < 0.05, **p < 0.01, ***p < 0.001 by Student’s *t*-test

Angiogenesis, especially that mediated by VEGF-A, is required for the increase in tumorigenicity of cells undergoing EMT. Interestingly, we noticed that the Bel/5-FU cells displayed a mesenchymal phenotype (Additional file 7) and the xenograft tumors injected with agomiR exhibited mesenchymal properties with an increase in N-Cadherin (N-Cad) and a decrease in E-Cadherin (E-Cad), but the injection of antagomiR resulted in opposite effects (Fig. 5a). These results indicated that miR-32-5p may contribute to multidrug resistance by mediating EMT. Additionally, we also observed that the HCC specimens of patients with higher level of miR-32-5p exhibit high N-Cad and low E-Cad expression (Fig. 5c). Therefore, we speculated that miR-32-5p induces multidrug resistance through EMT and angiogenesis.

To better elucidate the possible mechanism of miR-32-5p in multidrug resistance, Western blots were performed to detect the expression of N-Cad and E-Cad, and the results revealed that miR-32-5p mimics or siPTEN up-regulated N-Cad but down-regulated E-Cad, while miR-32-5p inhibitor or PTEN-expressing vector caused the opposite effects (Fig. 6a). We next evaluated the expression of Twist and Snail mRNA, both of which are downstream of the PI3K/Akt pathway and are important transcription factors in EMT. Real-time PCR showed that the expression of Twist and Snail mRNA increased with miR-32-5p mimics or siPTEN but decreased with miR-32-5p inhibitor or PTEN-expressing vector (Fig. 6c). As cells undergoing EMT gain invasion and migration abilities, wound healing and transwell assays were employed to reveal the role of miR-32-5p/PTEN/PI3K/Akt in EMT. As we expected, miR-32-5p mimics or siPTEN elevated invasion and migration abilities of the HCC cells, while miR-32-5p inhibitor or PTEN-expressing vector reduced these abilities (Fig. 6e, g, Additional file 8). Additionally, co-transfection of miR-32-5p mimics and PTEN-expressing vector or co-transfection of miR-32-5p inhibitor and siPTEN abolished the effects of miR-32-5p mimics or inhibitor alone, indicating that miR-32-5p targets PTEN activates the PI3K/Akt pathway to promote EMT process (Fig. 6e, g and Additional file 8).

**Fig. 7:** Exosomal miR-32-5p induces multidrug resistance in vitro and in vivo. **a** Schematic diagram of exosome extraction. **b** The sizes and numbers of exosomes were determined by a Delsa Nano Analyzer. **c** Western blots for the expression of the exosome markers Flotillin-1, TSG-101, and CD63. **d** miR-32-5p was overexpressed in exosomes from Bel/5-FU. **e** Real-time PCR for the expression of miR-32-5p in exosomes treated with ethanol and GW-4869. **f** Real-time PCR for the expression of miR-32-5p and PTEN in Bel7402 cells treated with PBS, exosomes from Bel/5-FU, mimics NC and mimics. **g** Exosomes from Bel/5-FU but not from Bel7402 induced multidrug resistance, and miR-32-5p inhibitor reversed resistance in Bel7402 cells. (**h** and **k**) Western blots for the expression of molecules of the PI3K/Akt pathway, E-cad and N-Cad in Bel7402 cells after treatment with PBS, exosomes from Bel7402 and Bel/5-FU; in Bel7402 cells into which miR-32-5p inhibitor or inhibitor NC was transferred after treatment with exosomes; and in Bel7402 cells transfected with miR-32-5p mimics and the respective NC. (**i** and **j**) Migration and invasion assay of Bel7402 cells after treatment with PBS, exosomes from Bel7402 and Bel/5-FU; Bel7402 cells into which miR-32-5p inhibitor or inhibitor NC was transferred after treatment with exosomes; and Bel7402 transfected with miR-32-5p mimics and the respective NC. (**l**) Growth curves of xenograft tumors derived from Bel7402 cells injected with exosomes and then treated with PBS or 5-FU. *n* = three independent experiments, *p < 0.05, **p < 0.01, ***p < 0.001 by Student’s *t*-test. (**m**) IHC staining for PTEN, p-Akt, p-mTOR, p-P70S6K, Ki67, N-Cad, E-Cad, and CD31 in xenograft tumors. Original magnification, 400×; scale bar, 25 μm. *p < 0.05, **p < 0.01, ***p < 0.001 by Student’s *t*-test. N-Cad, N-Cadherin; E-Cad, E-Cadherin; MVD, microvascular density. (**n**) Schematic diagram summarizing how exosomal miR-32-5p induces multidrug resistance via the PTEN/PI3K/Akt pathway through angiogenesis and EMT. Exo, exosome

Moreover, the level of VEGF in the supernatant of Bel7402 cells transfected with miR-32-5p mimics or siPTEN was significantly increased (*p* < 0.05); however, the level of VEGF in the supernatant of Bel/5-FU cells transfected with miR-32-5p inhibitor or PTEN-expressing vector was decreased (*p* < 0.05). Up- or down-regulation of PTEN reversed the effects of miR-32-5p mimics or inhibitor in VEGF expression (*p* < 0.05, Fig. 6d).

Then, we used WM to validate that miR-32-5p promoted angiogenesis and EMT by activating the PI3K/Akt pathway. Western blots showed that WM decreased the expression of N-Cad but increased the expression of E-Cad, indicating that WM suppressed EMT. However, the suppression of EMT was abolished by both the upregulation of miR-32-5p and the downregulation of PTEN (Fig. 6b, c, and Additional file 8). Moreover, the level of VEGF in the supernatant was also decreased after WM treatment but was increased with the transfection of miR-32-5p mimics or siPTEN (Fig. 6d). The invasion and migration abilities of the cells were dampened with the use of WM but recovered when the cells were transfected with miR-32-5p mimics or siPTEN (Fig. 6f, g and Additional file 8).

### Exosomal miR-32-5p leads to multidrug resistance

Thus, we proved that miR-32-5p confers multidrug resistance by activating the PI3K/Akt pathway and undergoing EMT and angiogenesis; however, how miR-32-5p transforms sensitive cells to resistant cells remains puzzling.

Exosomes derived from resistant cell lines can transfer oncogenic miRs to sensitive cell lines, thereby inducing resistance to chemodrugs. We performed ultracentrifugation to isolated exosomes from the resistant cell line Bel/5-FU and the sensitive cell line Bel7402 (as shown in Fig. 7a). Nano Analyzer was used to measure the size of the exosome and to further confirm the presence and purity of the exosomes. Exosome biomarkers, such as CD63, TSG-101 and Flotillin-1, were also examined to further verify the presence of exosomes (Fig. 7b and c). We used the exosomes from Bel7402 as a control and found that miR-32-5p was the most overexpressed miR in the exosomes from Bel/5-FU (Fig. 7d). The treatment of Bel/5-FU with GW4869, an inhibitor of the secretion of exosomes from cells, resulted in a reduction in the quantity of exosomes (Fig. 7b and c) as well as miR-32-5p (Fig. 7e). To exclude exosome transfer or stimulation by exosome treatment, we treated Bel7402 with the exosomes from Bel7402 and noted that the expression levels of miR-32-5p or PTEN did not change significantly compared with those in Bel7402 treated with PBS (Fig. 7f). Moreover, the IC50 of 5-FU, OXA, GEM, and sorafenib between Bel7402 treated with PBS and Bel7402 treated with exosomes from Bel7402 did not have significant difference (Fig. 7g). The expression of miR-32-5p in Bel7402 treated with exosomes from Bel/5-FU was higher than that in Bel7402 transfected with miR-32-5p mimics: the fold-change was 2.1 and 1.6, respectively, compared with the expression of miR-32-5p in Bel7402 treated with PBS. Meanwhile, the expression of PTEN mRNA was almost the same in Bel7402 treated with exosomes from Bel/5-FU and in Bel7402 transfected with miR-32-5p mimics (Fig. 7f). Moreover, exosomes from Bel/5-FU have similar effects to those of miR-32-5p mimics: MTT assay indicated that the IC50 of 5-FU, OXA, GEM, and sorafenib in Bel7402 increased after the transfection of exosomes from Bel/5-FU as well as miR-32-5p mimics (Fig. 7g); and Western blots showed that PTEN decreased but phosphorylated-mTOR, P70S6K, and Akt increased after the introduction of exosomes from Bel/5-FU, compared with the levels in Bel7402 treated with PBS and exosomes from Bel7402 (Fig. 7h). miR-32-5p inhibitor was used to confirm the role of exosomal miR-32-5p in inducing multidrug resistance. MTT assay and Western blots revealed miR-32-5p inhibitor reverses the effects of exosome from Bel/5-FU (Fig. 7g and h). These results indicate that exosomes derived from Bel/5-FU, but not from Bel7402, can transfer miR-32-5p into Bel7402, leading to an increase in miR-32-5p, a decrease in PTEN and activation of the PI3K/Akt pathway, and finally induces multidrug resistance.

Transwell and wound healing assays were conducted to investigate the effects of exosomes from Bel/5-FU, and the results showed that exosomes from Bel/5-FU but not from Bel7402 enhanced the invasion and migration abilities of Bel7402 and that exosomal miR-32-5p was the main cause of enhancement (Fig. 7i and j, Additional file 9). Western blots for N-Cad and E-Cad further confirmed the results of the invasion and migration experiments (Fig. 7k).

In vivo experiments suggest that exosomes from Bel/5-FU can confer 5-FU resistance (Fig. 7l and Additional file 10). Moreover, IHC of xenograft tumor specimens revealed that the PI3K/Akt pathway was activated upon exosome treatment. EMT and angiogenesis biomarkers also indicated that tumors treated with exosomes underwent EMT and angiogenesis (Fig. 7m).

In conclusion, we demonstrated that miR-32-5p is delivered to sensitive cells from resistant cells by exosomes, activates the PI3K/Akt pathway, and induces multidrug resistance by modulating angiogenesis and EMT (Fig. 2n).

## Discussion

In this study, we for the first time demonstrated miR-32-5p is delivered to sensitive cells from resistant cells by exosome, activates the PI3K/Akt pathway and induces multidrug resistance by modulating angiogenesis and EMT (Fig. 7n).

Previous studies from our group and others suggested that the loss of PTEN or reduced expression of PTEN leads to prolonged activation of the PI3K/Akt pathway, resulting in carcinogenesis [30, 34] as well as treatment resistance [4].

The PI3K/Akt pathway has been regarded as a molecular “crutch” for cells to escape death [35]. As we have verified miR-32-5p directly targets PTEN and activated the PI3K/Akt pathway, we decided to further investigate the underlying mechanisms of the miR-32-5p/PTEN/PI3K/Akt in inducing multidrug resistance. Contradictory to previous reports that the PI3K/Akt pathway promotes tumorigenesis or treatment resistance by inhibiting apoptosis, no significant changes in cell apoptosis were observed after the miR-32-5p intervention. Thus, we wondered whether the miR-32-5p/PTEN/PI3K/Akt pathway contributes to multidrug resistance through other mechanisms.

The tumor microenvironment, rather than the tumor cells directly, modulate the sensitivity of cells to anti-tumor therapies [36]. Vecchione et al. [33] found that miR-484 was associated with chemoresistance in ovarian cancer and determined that the sensitive phenotype is a result of modulation of the tumor vasculature through the regulation of the VEGFB and VEGFR2 pathways, rather than through the inhibition of apoptosis. Moreover, Wilson [37] pointed out that crosstalk between vasculature and tumor cells can be exploited to improve the efficacy of chemotherapy and radiation. Coincidently, we have previously demonstrated that the C2 domain of PTEN leads to tumor suppression through angiogenesis rather than by apoptosis [30]. Dong et al. [38] reported that loss of PTEN activated the PI3K/Akt pathway and STAT3, leading to increasing of VEGF. Based on these, we decided to determine if multidrug resistance is mediated by angiogenesis via the miR-32-5p/PTEN/PI3K/Akt pathway. As expected, we noticed an increased production of VEGF in tumor tissues from xenograft nude mice, as well as an elevated expression of CD31, an endothelial cell marker with the up-regulation of miR-32-5p. Furthermore, in vitro experiments show that VEGF secretion in the supernatant of cultured cell line increases with the activation of the miR-32-5p/PTEN/PI3K/Akt, but decreases with inhibition of the miR-32-5p/PTEN/PI3K/Akt, indicating the function of the miR-32-5p/PTEN/PI3K/Akt in VEGF secretion.

Angiogenesis, especially that mediated by VEGF-A, is required for the increase in tumorigenicity of cells undergoing EMT. Bu et al. [39] observed that PD-1 therapy-resistant melanoma patients display distinct signatures of up-regulated genes involved in angiogenesis and EMT, indicating that EMT accompanied with angiogenesis plays a vital role in the incidence of treatment resistance in cancer. Additionally, Fantozzi et al. [40] demonstrated a connection between VEGF-A-induced angiogenesis and EMT in breast cancer. In accordance with previous reports that chemoresistant cell lines often exhibit phenotypic changes consistent with EMT, we also noticed that the multidrug resistant cell line Bel/5-FU displays mesenchymal properties, with spindle-cell shape, loss of polarity, intercellular separation, and pseudopodia formation. Due to the significance of the PI3K/Akt pathway in the acquisition of resistance in cells to chemotherapeutic drugs and sorafenib, we assessed N-cad and E-Cad, the main criteria for EMT [41] in miR-32-5p up- and down-regulated cell lines as well as in xenograft tumors and found that the ectopic expression of miR-32-5p promoted mesenchymal but inhibited epithelial properties both in vitro and in vivo. We also demonstrated that Twist and Snail, both of which are important transcriptional factors of EMT, are regulated by the miR-32-5p/PTEN/PI3K/Akt. Up-regulated expression of Twist, a highly conserved bHLH transcription factor that is known to promote EMT, also promotes tumor angiogenesis [42]. Moreover, Snail1 has been proven to be regulated by the VEGF-A receptor to promote EMT [43]. These results further confirmed the interaction between angiogenesis and EMT.

In the end, we aim to find out the mechanisms underlying the transformation from sensitive cell line to multidrug resistant cell line. Various studies have already described the signaling pathways involved in the role of EVs in “educating” the cancer cell protrusive activity, motility, and metastasis. Cancer-derived exosomes are an important mediator of intercellular signaling and EMT, with resultant transformation of cancer cells to a more aggressive phenotype [44]. Importantly, the ability of exosomes shed by tumor drug-resistant cells to transfer the resistant phenotype to drug-sensitive cells has also been indicated as an important mechanism for “dissemination” of drug resistance, mainly through transferring of drug-efflux pumps and miRNAs. In our research, after estimating the regulation of miR-32-5p/PTEN/PI3K/Akt in multidrug resistance, we found out the exosomes delivered miR-32-5p from resistant cells to sensitive cells, and further activate the PI3K/Akt pathway in the sensitive cells and to “educate” the sensitive cells become multidrug resistant. In our point of view, long-term exposure of 5-FU upregulates miR-32-5p, elevated miR-32-5p is capsulated into exosomes and then is transferred to the sensitive cell, afterward, the sensitive cells receive miR-32-5p and activate the PI3K/Akt pathway and finally became resistant to multidrug.

In conclusion, our study is the first to demonstrate the miR-32-5p delivered by exosomes from resistant cells, activates the PI3K/Akt pathway and leads to multidrug resistance in HCC via angiogenesis and EMT.

## Conclusion

Our study demonstrated that the multidrug-resistant cells deliver miR-32-5p to sensitive cell by exosomes and activates the PI3K/Akt pathway to further induce multidrug resistance by modulating angiogenesis and EMT.

## Additional files

Additional file 1: miR-32-5p interference and sequences of PTEN siRNA. (DOCX 14 kb)

Additional file 2: Sequences of specific primers (DOCX 14 kb)

Additional file 3: Predicted binding sites of miR-32-5p, miR-21-5p, miR-19-3p, miR-92-3p, miR-486-5p and PTEN 3’-UTR (TIFF 1854 kb)

Additional file 4: miR-32-5p is conserved in different species. Cfa, dog; mmu, mouse; rno, rat; gga, chicken; mml, rhesus; mdo, opossum; bta, cow; ptr, chimpanzee. (TIFF 2183 kb)

Additional file 5: miR-32-5p promotes multidrug resistance in vivo. (A) Schematic diagram of the in vivo experiments. The red dots represent the injection of agomiR, agomiR NC, antagomiR, and antagomiR NC; injections started on the 2nd week and continued twice per week for three weeks. The green arrows represent injections of 5-FU or 0.9%NS; injection started on the 3rd week and continued once a week for three weeks. (B) Tumors formed from Bel7402 cells injected with agomiR and Bel/5-FU cells injected with antagomiR. (TIFF 12931 kb)

Additional file 6: miR-32-5p does not affect apoptosis. (A) Flow cytometric analysis of apoptosis rate in Bel7402 cells transfected with miR-32-5p mimics, Bel/5-FU cells transfected with miR-32-5p inhibitor and the respective NC. (B) Apoptosis rate in Bel7402 cells transfected with miR-32-5p mimics, Bel/5-FU cells transfected with miR-32-5p inhibitor and the respective NC. n = three independent experiments, by Student’s *t*-test. (C) Western blots for caspase 3 in Bel7402 cells transfected with miR-32-5p mimics, Bel/5-FU cells transfected with miR-32-5p inhibitor and the respective NC. The expression of caspase 3 is normalized to the level of the corresponding internal control β-actin. (TIFF 8394 kb)

Additional file 7: Bel/5-FU cell line exhibits mesenchymal properties. The left panel is the representative image of sensitive cell line Bel7402, and the right panel is the representative image of multidrug-resistant cell line Bel/5-FU. Original magnification, 400 × (TIFF 6057 kb)

Additional file 8: Wound healing assay to detect the migration ability. (A-C) Wound healing assay of Bel7402 and Bel/5-FU cell lines transfected with miR-32-5p mimics, inhibitor, siPTEN or PTEN-expressing vector, co-transfected with miR-32-5p mimics and PTEN-expressing vector or miR-32-5p inhibitor and siPTEN, and WM-treated Bel/5-FU cell lines transfected with miR-32-5p mimics or siPTEN. Original magnification, 200 × (TIFF 4093 kb)

Additional file 9: Wound healing assay to detect the migration ability after exosome treatment in Bel/5-FU. Original magnification, 200 × (TIFF 8930 kb)

Additional file 10: Exosomal miR-32-5p promotes 5-FU resistance in vivo. Tumors formed from Bel7402 cells injected with PBS and exosomes from Bel/5-FU cells treated with 0.9%NS or 5-FU (TIFF 4545 kb)

## Abbreviations

0.9%NS: 0.9% normal saline
5-FU: 5-fluorouracil
AJCC: American Joint Committee on Cancer
E-Cad: E-Cadherin
ELISA: Enzyme-linked immunosorbent assay
EMT: Epithelial to mesenchymal transition.
EXO: Exosome
FFPE: Formalin-fixed, paraffin-embedded
FBS: Fetal bovine serum
GEM: Gemcitabine
HCC: Hepatocellular carcinoma
IHC: Immunohistochemistry
miR: microRNA
MTT: 3-(4,5-dimethyl-2-thiazolyl)-2,5-diphenyl-2H-tetrazolium bromide
MuT: Mutant type
MVD: Microvascular density
N-Cad: N-Cadherin
NC: Negative control
OS: Overall survival
OXA: Oxaliplatin
PFS: Progression free survival
TCGA: The Cancer Genome Altas
WM: Wortmannin
WT: Wild type
